RETRACTED

# Long Noncoding RNA Zinc Finger Antisense 1 Affects Glucocorticoid-Induced Osteonecrosis of the Femoral Head by Performing as a ceRNA for MicroRNA-124-3p and Accelerating Transforming Growth Factor Type III Receptor

**DOI:** 10.1155/2022/4487864

**Published:** 2022-07-18

**Authors:** Xiao Yong Lan, YiPin Xiong, HaiPing Ma, LingFeng Zou, Zhen Yuan, YuHong Xiao

**Affiliations:** ^1^Department of Rehabilitation Medicine, Second Affiliated Hospital of Nanchang University, Nanchang City, Jiangxi Province 330008, China; ^2^Department of Ultrasound (Musculoskeletal Ultrasound), Second Affiliated Hospital of Nanchang University, Nanchang City, Jiangxi Province 330008, China; ^3^Department of Nursing, Second Affiliated Hospital of Nanchang University, Nanchang City, Jiangxi Province 330008, China

## Abstract

In recent years, plentiful studies have uncovered the long noncoding RNA's (lncRNA's) momentous functions in osteonecrosis of the femoral head (ONFH), but the specific mechanism has not been fully illustrated. The study was to figure out lncRNA Zinc finger antisense 1 (LncZFAS1)'s biological function and its latent downstream molecular mechanism in glucocorticoid- (GC-) induced ONFH. The results manifested LncZFAS1 and transforming growth factor type III receptor (TGFBR3) were elevated, while microRNA- (miR-) 124-3p was reduced in ONFH tissues and cells. Knockdown LncZFA1 reduced rat femoral cell apoptosis, perfected bone microstructure and bone density, and accelerated osteogenic proteins bone morphogenetic protein- (BMP-) 9, BMP-3, and osteocalcin. In vitro studies manifested knockdown LncZFAS1 prevented GC-induced reduction in osteoblast advancement with facilitating osteoblast calcification capacity, ALP activity, and osteogenic proteins. Elevation of LncZFAS1 further aggravated GC-induced osteoblast injury, but this effect was turned around by enhancement of miR-124-3p or knockdown of TGFBR3. Mechanistically, LncZFAS1 performed as a sponge for miR-124-3p to mediate TGFBR3 expression to motivate GC-induced ONFH. All in all, the results of this study indicate the LncZFAS1/miR-124-3p/TGFBR3 axis is supposed to be a latent therapeutic molecular target for GC-induced ONFH.

## 1. Introduction

Osteonecrosis of the femoral head (ONFH) is a familiar orthopedic disease frequently taking place after glucocorticoid (GC) therapy [1]. GC has been reported to stimulate ONFH pathogenesis by directly damaging blood vessels and declining blood supply to the femoral head, as well as by motivating oxidative stress to induce apoptosis in BMSCs [2]. These changes can result in disruption of the blood supply and disturbance of the coagulation and fibrinolytic systems, causing the collapse of the femoral head [3]. Currently, once GC-induced ONFH occurs, there is no effective cure to turn around its development [4]. Therefore, there is an urgent need to develop effective measures to enhance BMSC osteogenic differentiation and angiogenesis to prevent GC-induced ONFH's presence. Long noncoding RNA (lncRNA) is a noncoding RNA, which participates in diversified physiological and pathological processes and performs also as a regulator in all kinds of human diseases [5–9].

microRNAs (miRNAs), a class of brief endogenous noncoding RNAs, modulate posttranscriptional gene expression by combining with the 3′-untranslated region (UTR) of target RNAs and participate in diversified cellular biological processes, covering growth, cell cycle, migration, differentiation, and apoptosis [10]. Plentiful studies have manifested miRNA dysregulation is the crux to the occurrence of numerous diseases, like various bone diseases [11, 12]. Former studies have clarified miR-124-3p is elevated in the serum of patients with distal tibial metaphysis fractures and mediates fracture healing by reducing apoptosis by repressing bone morphogenetic protein (BMP) 6 [13]. Another study clarifies miR-124-3p is reduced in osteoarthritis, and elevation of miR-124-3p perfects osteoarthritis by suppressing inflammation by depressing NF-*κ*B and IL-6 [14]. However, the expression and function of miR-124-3p in GC-induced ONFH remain unknown. This refers to noncoding RNA with a length greater than 200 nucleotides. lncRNA has a very important regulatory function and almost participates in various biological processes and pathways. It is closely related to the occurrence and development of various diseases, so it has become a research hotspot and focus in the past few years and the future. For the human genome, the number of lncRNAs produced is much more than the number of coding RNA. At present, except for a few lncRNAs whose functions are relatively clear, the functions of most lncRNAs are unknown. It is very worthy of further study.

RETRACTED

In the present study, it was speculated that LcnZFAS1 was supposed to be involved in ONFH's development. ONFH *in vitro* and *in vivo* models were established by dexamethasone (DEX) treatment. The biological function of LncZFAS1 in ONFH was figured out by gene knockdown or elevation. Moreover, through functional rescue experiments, it was further testified that LncZFAS1 influences ONFH's development via downstream signaling pathway miR-124-3p/transforming growth factor type III receptor (TGFBR3).

## 2. Materials and Methods

### 2.1. Clinical Sample Collection

From April 2016 to March 2019, collection of femoral head tissue was from 38 ONFH patients (23 males and 15 females, age of 53 ± 11 years) admitted to the Department of Osteoarthritis and Joint Surgery of Second Affiliated Hospital of Nanchang University. Meanwhile, collection of the femoral head tissues of 16 patients (10 males and 6 females, age of 48 ± 9 years) undergoing total hip arthroplasty with femoral neck fracture was as controls. No clear differences were presented in gender, age, and body mass index of the patients in the two groups (*P* > 0.05). Obtaining written informed consent was from all subjects prior to the study. The protocol of this study was ratified by the Ethics Committee of Second Affiliated Hospital of Nanchang University and complies with the ethical principles of medical research in the *Declaration of Helsinki*.

### 2.2. ONFH Animal Model

Obtaining 40 8-week-old male Sprague Dawley rats (weight of 200-250 g) was from the Experimental Animal Center of Second Affiliated Hospital of Nanchang University, and feeding the animals was in a standard experimental environment (12 h light cycle, at 24 ± 2°C, 50%-60% humidity), with free access to food and water. After one week of adaptive feeding, casual assignation of animals was into 3 groups (*n* = 10): the control, the ONFH, and the Lv-sh-negative control (NC)/ZFAS1. In the ONFH, establishment of the ONFH model was by intramuscular injection of DEX (Sigma-Aldrich, 5 mg/kg) twice a week for 6 weeks. Injection of the control was with the same dose of normal saline. After establishment of the ONFH model in the Lv-sh-NC/ZFAS1, application of a number 33 needle (Hamilton Company, Bonaduz, Switzerland) and a 25 *μ*l CASTIGHT syringe (Hamilton Company) was to inject short hairpin RNA adenoviral vector targeting LncZFAS1 or NC vector (50 *μ*L each, once every 2 d for 3 weeks) into the distal femur of the rat medullary cavity. Subsequently, euthanasia of the rats and collection of femoral tissue for subsequent experiments were conducted.

### 2.3. Hematoxylin-Eosin (HE) Staining

Collection and fixation of distal femurs in 10% neutral formaldehyde were conducted. Subsequently, removing the femurs, decalcification in 10% ethylene diamine tetra-acetic acid solution (pH 7.4), embedding in paraffin, then cutting into sections with 5 *μ*m thickness, and HE staining were implemented. Observation of histopathological changes was under a fluorescence microscope (Olympus IX53; Olympus Corporation). Measurement of relative damage levels in each group was by cortical area, and analysis was conducted applying the ImageJ software (version 1.48; National Institutes of Health).

### 2.4. Immunochemistry

Dewaxing and dehydration of sections and immersing in 3% H_2_O_2_ to inactivate endogenous enzymes were conducted. After adding 5% bovine serum albumin, supplement of the sections was with primary antibodies BMP-3 (ab134724), BMP-9 (ab35088), and OCN (ab93876) (all Abcam). Subsequently, addition of horseradish peroxidase- (HRP-) labeled secondary antibody to the sections, incubation, addition of streptavidin-biotin complex, and incubation were conducted. Application of diaminobenzidine (DAB) was for color development. Counterstaining of sections was with hematoxylin, dehydration, and permeabilization with xylene, and seal with neutral balsam was conducted.

RETRACTED

### 2.5. Dual Energy X-Ray Absorption (DXA) Analysis

DXA measurements were performed applying a Hologic DXA device (Hologic Discovery W 81507; Hologic, Inc.) to scan and measure the bone mineral density (BMD) of each rat. Results were manifested as grams of mineral content per square centimeter of bone area (g/cm^2^).

### 2.6. Terminal Deoxynucleotidyl Transferase-Mediated dUTP-Biotin Nick End Labeling (TUNEL) Staining

Detection of apoptotic cells in apoptotic femoral tissue was conducted applying a TUNEL assay and an in situ cell death detection kit (Roche Diagnostics, Mannheim, Germany) in the light of the manufacturer's instructions. Briefly, after routine dewaxing and treatment with H_2_O_2_ (3%), detachment of sections was with proteinase K (pH 7.4) and incubation of the reaction mixture (1 : 40) was conducted. Then, detection of bound fluorescein was with horseradish peroxidase, followed by staining with DAB. Assessment of Brown nuclei was as positive apoptotic cells.

1. For one-sided tolerances

(1) $$\begin{array}{c} Z=\frac{\bar{\bar{X}}-\text{LSL}}{{\hat{\sigma }}_{\bar{R}/d2}}, \end{array}$$

where LSL is defined as the lower instructional target limit, $\bar{\bar{X}}$ is the process mean, and $\hat{\sigma }$ is the process deviation, calculated from *R*/*d*_2_.

(2) For the two-way tolerance, the percentage of exceeding the upper and lower normative limits are calculated, respectively. zmin can also be converted into a capacity index*C*_*pk*_ as defined in the following equation.

(2) $$\begin{array}{c} Z_{\text{USL}}=\frac{\text{USL}-\bar{\bar{X}}}{{\hat{\sigma }}_{\bar{R}/d2}},\\ Z_{\text{LSL}}=\frac{\bar{\bar{X}}-\text{USL}}{{\hat{\sigma }}_{\bar{R}/d2}}. \end{array}$$

### 2.7. Cell Culture

The murine osteoblast cell line MC3T3-E1 (ATCC® CRL-2594) was from the American Type Culture Collection. Cells were grown in *α*-minimal essential medium (*α*-MEM) covering 10% fetal bovine serum (Gibco; Thermo Fisher Scientific, Inc.), 100 U/ml penicillin, and 100 *μ*g/ml streptomycin (Gibco; Thermo Fisher Scientific, Inc.) and maintained at 37°C in a humidified environment with 5% carbon dioxide, with changing the medium every 2 d. Subsequently, treatment of cells was with different concentrations of DEX.

RETRACTED

### 2.8. Cell Transfection

Purchase of small interfering RNA targeting LncZFAS1 and TGFBR3 with NCs (si-ZFAS1/TGFBR3/NC) and elevation plasmids (oe-ZFAS1/TGFBR3/NC) and miR-124-3p-mimic/inhibitor and NCs was from GenePharma (Shanghai, China). To alter gene expression, transient transfection of the above plasmids or oligonucleotides was into MC3T3-E1 cells applying Lipofectamine 2000 (Invitrogen), and assessment of transfection efficiency was conducted by RT-qPCR 48 h later.

### 2.9. Alizarin Red Staining

Detection of calcium nodule formation was by Alizarin red staining. Detachment and seeding of osteoblasts in 24-well plates were conducted. Addition of paraformaldehyde (5%, 500 *μ*l) and alizarin (200 *μ*l) was to the medium sequentially, and photomicrographs of calcium nodules were taken.

### 2.10. Alkaline Phosphatase (ALP) Staining

Seeding of MC3T3-E1 cells (1.2 × 10^4^ cells/well) was in 6-well plates. *In vitro* and *in vivo* determination of ALP activity was performed applying an ALP staining kit (Thermo Fisher Scientific, Inc.) following the manufacturer's protocol. Subsequently, measurement of OD values was at 540 nm applying a microplate reader (Infinite™ M2000; Tecan Group, Ltd.), and observation and collection of images were implemented under an inverted fluorescence microscope (Olympus Corporation).

### 2.11. Cell Counting Kit- (CCK-) 8 Detection of Cell Viability

Seeding of DEX or transfected cells was in 96-well plates (5 × 10^3^ cells/well). Treatment of cells was with 10 *μ*l CCK-8 reagent per well and incubation was conducted. Finally, measurement of absorbance was at 450 nm on a microplate reader (Thermo Fisher Scientific, Inc.).

### 2.12. Reverse Transcription Quantitative Polymerase Chain Reaction (RT-qPCR)

Extraction of total RNA from tissues and cells was with TRIzol reagent (TaKaRa Bio, Inc.) in the light of the manufacturer's protocol. Reverse transcription of total RNA (5 *μ*g) was into complementary DNA applying the PrimeScript RT kit (ELK Biotechnology). Performing RT-qPCR was in triplicate applying the following protocol. Performing PCR was on an ABI 7500 Real-Time PCR System (ABI, NY, USA) applying the SYBR premix Ex Taq II kit (ELK Biotechnology). Obtaining primers was from Shanghai Gene Pharmaceutical Co., Ltd. The primer sequence was manifested in Table 1. Quantification of results was conducted applying the ^2-*ΔΔ*Cq^ method. Application of an internal reference gene (U6 or glyceraldehyde-3-phosphate dehydrogenase (GAPDH)) was for normalization.

### 2.13. Western Blot

Extraction of total proteins in tissues and cells was by radioimmunoprecipitation, and determination of protein concentrations was implemented applying a bicinchoninic acid kit (Wuhan Bost Biotechnology Co., Ltd., Hubei, China). Addition of 30 *μ*g sample to each well, 10% polyacrylamide gel electrophoresis, electroblot onto polyvinylidene fluoride membrane, and blocking with 5% skimmed milk were conducted. Next, incubation of membranes was with the following primary antibodies BMP-3 (ab134724), BMP-9 (ab35088) and OCN (ab93876) (all Abcam), TGFBR3 (2519), GAPDH (2118) (both Cell Signaling Technology), and goat anti-rabbit HRP-conjugated secondary antibody (Shanghai Miaotong Biotechnology Co., Ltd., China). Visualization of all specific bands was with the electrogenerated chemiluminescence system kit (Pierce Biotechnology, Beijing, China), and detection of the density values was with the ImageJ software (NIH, Bethesda, MD, United States). GAPDH served as an internal reference protein.

RETRACTED

### 2.14. The Luciferase Activity Assay

Construction of Wild-type and mutant sequences of LncZFAS1 and TGFBR3 (WT/MUT-LncZFAS1 and WT/MUT-TGFBR3) was implemented applying the partial sequence of LncZFAS1 covering the putative binding site of miR-124-3p and the TGFBR3 3′ UTR. Synthesis of these sequences was by Sangon Biotech, and clone into pmirGLO Dual-Luciferase miRNA target expression vector (Promega) was conducted. Cotransfection of the above vector was with miR-124-3p-mimic or mimic-NC into MC3T3-E1 cells applying Lipofectamine 2000 (Invitrogen) in the light of the manufacturer's instructions. Then, collection of cells was conducted, and quantification of the Firefly luciferase activity was implemented applying the Dual-Luciferase Reporter Assay System (Promega Corporation). Normalization of the data was to Renilla luciferase activity.

### 2.15. RNA-Binding Protein Immunoprecipitation (RIP) Assay

RIP assay was implemented to examine the relationship between genes. After lysis of cells with IP buffer (Thermo Fisher Scientific), centrifugation of the cell lysates and collection of the supernatant were conducted. Subsequently, addition of 20 *μ*L protein magnetic beads (Millipore, Darmstadt, Germany), incubation with lysate, and addition of anti-Ago2 antibody and IgG were conducted. Finally, purification of RNA was from magnetic beads applying TRIzol reagent, and detection of RNA enrichment was by RT-qPCR.

The purpose of this study is to investigate the effects of glucocorticoids (GCs) on chondrocytes and the protective effects of rifampicin on them. Methods: chondrocytes were isolated from the knee joint of SD rats, cultured and treated with different concentrations of dexamethasone (DEX). According to the principle of randomized control, they were divided into three groups: NS (CON) group, DEX group, and dex+rif group. The levels of reactive oxygen species (ROS) and the expression of parathyroid hormone (PTH)/parathyroid hormone-related peptide receptor (PTH1R) in chondrocytes were measured. The expression level of apoptosis-related proteins in chondrocytes was further studied by Western blot. Results after GC treatment: there was cavity cartilage abnormality in the subchondral area. Osteoclast activity increased. At the same time, ROS level and PTH1R expression increased after GC treatment. In the dex+rif group, rifampicin protected chondrocytes from DEX-induced apoptosis. Conclusion: the decrease of ROS production and PTH1R expression can make rifampicin reduce the apoptosis of DEX-treated chondrocytes. A large number of chondrocyte apoptosis may be the characteristic marker of early ONFH;

RETRACTED

### 2.16. Data Analysis

Application of GraphPad Prism 9.0 (GraphPad Software Inc., La Jolla, CA) was for all the above statistical analyses. Manifestation of the data was as mean ± standard deviation (SD). Application of unpaired Student's *t*-test was for comparisons between two groups, with one-way analysis of variance (ANOVA) and Tukey's post hoc test for multiple groups' comparisons. *P* < 0.05 emphasized obvious statistical meaning. All experiments in the research were carried out with at least three biological replicates.

## 3. Results

### 3.1. LncZFAS1 Is Elevated in ONFH

Detection of LncZFAS1 in ONFH patients was firstly implemented. As manifested in Figure 1(a), LncZFAS1 was elevated in the femoral tissue of ONFH patients vs. controls. Subsequently, through GC induction, the ONFH rat model was established. Meanwhile, it was clarified that the trabecular bone in the ONFH was small, scattered, and broken, with diffuse necrotic bone cells and elevated fibrous tissue in the bone (Figure 1(b)). DXA analysis manifested the BMD of the ONFH was clearly reduced vs. the control (Figure 1(c)). Additionally, the femoral ALP in the ONFH was memorably reduced vs. the control (Figure 1(d)). It came out vs. the control, the apoptosis rate of osteocytes in the femur of the ONFH was distinctly elevated (Figures 1(d) and 1(e)). Subsequently, osteogenic proteins BMP-9, BMP-3, and OCN were examined. The results manifested BMP-9, BMP-3, and OCN in the femur of the ONFH were apparently declined vs. the control (Figure 1(f)). These results manifested that it successfully established the ONFH model. Subsequently, detection of LncZFAS1 in ONFH rats was conducted. As clarified in Figure 1(g), LncZFAS1 was elevated in the ONFH vs. the control.

RETRACTED

### 3.2. Knockdown LncZFAS1 Perfects ONFH in Rats

Subsequently, it explored the effect of knocking down LncZFAS1 on ONFH through loss-of-function experiments. LncZFAS1 was knocked down by delivering a shRNA adenoviral vector targeting LncZFAS1 into the femur, and the knockdown efficiency was tested (Figure 2(a)). It turned out after repressing LncZFAS that the trabecular bone was clearly enlarged, the fracture phenomenon and diffuse necrotic bone cells were reduced, and the fibrous tissue in the bone was memorably reduced (Figure 2(b)). Furthermore, knockdown of LncZFAS1 elevated the BMD of the femur (Figure 2(c)). It was clarified that knockdown LncZFAS1 elevated ALP in the femur (Figure 2(d)). Meanwhile, the apoptotic rate of osteocytes in the femur was clearly reduced after LncZFAS1 knockdown (Figures 2(d) and 2(e)). Moreover, knockdown LncZFAS1 motivated BMP-9, BMP-3, and OCN in the femur (Figures 2(e) and 2(f)). These results suggested knockdown of LncZFAS1 effectively ameliorated ONFH in rats.

### 3.3. Knockdown LncZFAS1 Motivates Osteoblast Viability and Bone Formation

Next, it explored the effect of LncZFAS1 on GC-induced osteoblast injury *in vitro*. First treatment of the murine osteoblast cell line MC3T3-E1 cells was with different concentrations of DEX. As manifested in Figure 3(a), DEX dose-dependently restrained cell viability, and the cell viability of MC3T3-E1 cells was reduced to 43.74 ± 3.69% after 5 *μ*M DEX treatment. Subsequently, it knocked down LncZFAS1 in MC3T3-E1 cells by transfecting siRNA targeting LncZFAS1 (Figure 3(b)). It came out MC3T3-E1 cell viability was effectively restored after knockdown of LncZFAS1 (Figure 3(c)). Meanwhile, DEX treatment motivated apoptosis in MC3T3-E1 cells, whereas knockdown of LncZFAS1 attenuated this effect (Figure 3(d)). Moreover, DEX treatment reduced calcified nodules and ALP activity in MC3T3-E1 cells, while knockdown of LncZFAS1 alleviated this phenomenon (Figures 3(e) and 3(f)). DEX treatment declined BMP-9, BMP-3, and OCN in MC3T3-E1 cells, whereas knockdown of LncZFAS1 memorably restored these three proteins (Figure 3(g)). These results suggested knockdown LncZFAS1 motivated osteoblast viability and bone formation.

### 3.4. LncZFAS1 Competitively Adsorbs miR-124-3p

Next, exploration of LncZFAS1's downstream miRNA was conducted. Via Bioinformatics website https://cm.jefferson.edu/rna22/, it was forecast that miR-124-3p was supposed to be a latent target of LncZFAS1, and they had latent binding sites (Figure 4(a)), and miR-124-3p has been found to be a momentous member of femoral head dysfunction [15]. In the present study, it was discovered that miR-124-3p was reduced in both GC-induced femoral tissue and osteoblasts, but after knockdown of LncZFAS1, miR-124-3p both *in vivo* and *in vitro* models was recovered to varying degrees (Figures 4(b) and 4(c)). Subsequently, their targeted link was further checked. As clarified in Figure 4(d), luciferase activity was reduced after cotransfection of WT-LncZFAS1 and miR-124-3p-mimic, but cotransfection of MUT-LncZFAS1 with miR-124-3p-mimic had no effect on luciferase activity.  Figure 4(e) manifested enriched LncZFAS1 and miR-124-3p were presented in the Ago2 vs. the IgG. These results clarified LncZFAS1 competitively adsorbed miR-124-3p.

RETRACTED

### 3.5. LncZFAS1 Influences Osteoblast Viability and Bone Formation by Modulating miR-124-3p

Subsequently, oe-LncZFAS1 and miR-124-3p-mimic were cotransfected into MC3T3-E1 cells. It came out elevation of LncZFAS1 declined miR-124-3p, but cotransfection of miR-124-3p-mimic restored miR-124-3p (Figure 5(a)). Meanwhile, elevation of LncZFAS1 further reduced cell viability, while concurrent enhancement of miR-124-3p prevented this effect (Figure 5(b)). It came out elevation of LncZFAS1 motivated apoptosis, but at the same time, enhancement of miR-124-3p alleviated it (Figure 5(c)). Additionally, strengthening LncZFAS1 reduced the number of calcified nodules and ALP activity in cells, but concurrent elevation of miR-124-3p memorably restored them (Figures 5(d) and 5(e)). Furthermore, it turned out elevation of LncZFAS1 restrained BMP-9, BMP-3, and OCN in cells, while concurrent elevation of miR-124-3p reversed this effect (Figure 5(f)). These results suggested LncZFAS1 influenced osteoblast activity and bone formation by modulating miR-124-3p.

### 3.6. miR-124-3p Targets TGFBR3

The assumed binding site of TGFBR3 with miR-124-3p was discovered via bioinformatics website forecast (Figure 6(a)). Elevated TGFBR3 was discovered in ONFH patients as well as GC-induced ONFH rats and osteoblasts, while knockdown or elevation of miR-124-3p facilitated and repressed TGFBR3 in osteoblasts, respectively (Figures 6(b) and 6(c)). Additionally, it came out the luciferase activity was reduced by the cotransfection of WT-TGFBR3 and miR-124-3p-mimic, while mut-TGFBR3 and miR-124-3P-mimic had no effect on luciferase activity (Figure 6(d)). Moreover, TGFBR3 and miR-124-3p were distinctly enriched in the Ago2 vs. the IgG (Figure 6(e)). These results clarified miR-124-3p targeted TGFBR3.

### 3.7. Elevation of TGFBR3 Represses Osteoblast Viability and Bone Formation

Next, it examined the effect of TGFBR3 on GC-treated osteoblasts. The elevation plasmid targeting TGFBR3 was transfected into MC3T3-E1 cells to upregulate TGFBR3 (Figure 7(a)). It came out upregulation of TGFBR3 further suppressed osteoblast viability but motivated apoptosis (Figures 7(b) and 7(c)). Meanwhile, upregulation further reduced osteoblast calcified nodule numbers and ALP activity (Figures 7(d) and 7(e)). Moreover, enhancing TGFBR3 suppressed BMP-9, BMP-3, and OCN in osteoblasts (Figure 7(f)). These results suggested elevation of TGFBR3 refrained osteoblast advancement with bone formation.

RETRACTED

### 3.8. GC Impacts Osteoblast Viability and Bone Formation by Modulating the LncZFAS1/miR-124-3p/TGFBR3 Axis

Subsequently, oe-LncZFAS1 and si-TGFBR3 were transfected in DEX-treated MC3T3-E1 cells to explore the role of LncZFAS1/miR-124-3p/TGFBR3. As manifested in Figure 8(a), transfection of oe-LncZFAS1 reduced miR-124-3p but accelerated TGFBR3, whereas cotransfection of si-TGFBR3 had no effect on miR-124-3p but turned around TGFBR3. Functional experiments clarified transfection of oe-LncZFAS1 repressed cell advancement with reduced the number of calcified nodules and ALP activity as well as BMP-9, BMP-3, and OCN expression, but these effects were turned around via cotransfection of si-TGFBR3 (Figures 8(b)–8(f)). These results suggested the LncZFAS1/miR-124-3p/TGFBR3 axis was a crucial pathway by which GC affect osteoblast viability and bone formation.

## 4. Discussion

GC is an extremely familiar cause of ONFH, and this complication takes place in up to 40% of young adults treated for GC [16]. Its main pathological feature is the progressive necrosis of bone cells and bone marrow, eventually resulting in structural changes or even complete collapse of the femoral head [17]. As a gene expression regulator, lncRNA has been confirmed to modulate the differentiation and formation of osteocytes and take on a momentous role in GC-induced ONFH [18]. In this study, it was found that LncZFAS1 was elevated in the femur tissue of ONFH patients, suggesting that LncZFAS1 might be involved in the occurrence of ONFH. *In vivo* animal experiments clarified LncZFAS1 was elevated in ONFH rats, and knockdown LncZFAS1 effectively repressed the development of ONFH in rats. Meanwhile, the results of *in vitro* experiments manifested knockdown LncZFAS1 motivated osteoblast advancement with bone formation. These results suggest LncZFAS1 may perform as a negative regulator of ONFH.

Osteoblast differentiation refers to the process by which relatively unspecialized cells acquire the features of osteoblasts, which are the major functional cells in bone formation and are responsible for the synthesis, secretion, and mineralization of bone matrix [19]. Osteogenic differentiation is a complex process involving multiple signaling pathways as well as cytokines, such as the BMP family [20]. BMPs are paracrine and autocrine growth factors participating in diversified biological processes and a member of the transforming growth factor beta superfamily that modulates bone mass, fracture risk, fracture repair, and osteoblastogenesis and motivates osteogenesis [21], where BMP-9 [22] and BMP-3 [23] are positive and negative regulators of osteogenesis, separately. One of the markers of osteoblast differentiation is osteocalcin (OCN), and high OCN forecasts elevated osteoblast differentiation [24]. Therefore, exploring the modulatory mechanism of osteogenic differentiation is helpful to develop new therapeutic strategies for GC-induced ONFH. Recently, elevated studies have manifested lncRNA takes on a momentous function in GC-induced ONFH's pathogenesis. For example, lncRNA AWPPH is downregulated in ONFH patient serum and represses ONFH development by motivating osteoblast differentiation by elevating Runx2 [25]. LncRNA HOTAIR is upregulated in ONFH patients and motivates ONFH development by targeting the miR-17-5p/SMAD7 axis to refrain BMSC proliferation and osteogenic differentiation [3]. In the present study, it was found that LncZFAS1 was elevated in the serum of ONFH patients. Meanwhile, it was also detected elevated LncZFAS1 in GC-induced ONFH *in vivo* and *in vitro* models. Subsequent loss-of-function experiments and *in vitro* experiments consistently confirmed knockdown LncZFAS1 restrained ONFH progression by accelerating osteoblast proliferation and differentiation. These results suggest knockdown LncZFAS1 takes on a protective role in GC-induced ONFH, and LncZFAS1 may offer as a latent target for ONFH therapy.

RETRACTED

It has been reported that lncRNA frequently modulates disease progression by controlling miRNAs [26]. In the present study, it was found that LncZFAS1 was negatively linked with miR-124-3p in GC-induced ONFH. It was found that LncZFAS1 had binding sites with miR-124-3p and further confirmed that miR-124-3p was the target of LncZFAS1. miR-124-3p has been reported to be a crucial member of steroid-induced femoral head necrosis dysfunction [15]. Additionally, some studies have shown that miR-124-3p is closely linked with the osteogenic differentiation of BMSCs. For example, in diabetic osteoporotic rats, miR-124-3p motivates BMSC osteogenesis by depressing the GSK-3*β*/*β*-catenin signaling pathway [27]. miR-124-3p constrains the osteogenic differentiation of BMSCs in osteoporosis through the IGF2BP1/Wnt/*β*-catenin axis [28]. However, miR-124-3p's function in GC-induced ONFH is uncertain. Here, it was originally found that miR-124-3p was reduced in both GC-induced femoral tissue and osteoblasts, and elevation of miR-124-3p reversed the repression of enhancement of LncZFAS1 on osteoblast proliferation and differentiation. This finding suggests LncZFAS1 modulates GC-induced ONFH development by acting as a sponge for miR-124-3p. Many studies have clarified miRNAs generally modulate various cellular biological processes by targeting and modulating target genes. For example, miR-542-3p targeting BMP-7 signaling restrains osteoblast proliferation, differentiation, and bone formation [29]. In the present study, it was demonstrated that miR-124-3p modulated osteoblast function by targeting TGFBR3.

RETRACTED

Transforming growth factor type III receptor (TGFBR3) is a coreceptor for diversified ligands of the transforming growth factor-*β* (TGF-*β*) family, and proteins of the TGF-*β* superfamily have a remarkable ability to induce cartilage and bone [30, 33, 34]. A previous study manifests TGFBR3 has been shown to be elevated in osteoblasts from patients with osteogenesis imperfecta [31]. Recent studies have shown TGFBR3 takes on an important role in the development of blood vessels and osteoblasts [32]. In the present study, it was found that TGFBR3 was upregulated in GC-induced ONFH, and elevation of TGFBR3 refrained osteoblast proliferation and bone formation. Functional experiments manifested knockdown of TGFBR3 could reverse the effect of upregulated LncZFAS1 on ONFH. These results suggested the LncZFAS1/miR-124-3p/TGFBR3 axis was a crucial pathway by which GCs affect osteoblast proliferation and bone formation.

## 5. Conclusion

Taken together, the results of the present study suggest LncZFAS1 affects GC-induced ONFH by regulating osteoblast proliferation and bone formation by upregulating TGFBR3 via regarding as a ceRNA of miR-124-3p. These data reveal the LncZFAS1/miR-124-3p/TGFBR3 axis may offer as a latent therapeutic target for GC-induced ONFH.

## Figures and Tables

**Figure 1:** LncZFAS1 is elevated in ONFH. (a) RT-qPCR to detect LncZFAS1 in ONFH patients; (b) HE staining to detect the pathological changes of ONFH rat femur; (c) DXA analysis to detect ONFH rat femur BMD; (d) RT-qPCR to detect ALP in ONFH rat femur; (e) TUNEL staining to detect the apoptosis of ONFH rat femur osteocytes; (f) immunohistochemistry to detect BMP-3, BMP-9, and OCN in ONFH rat femur; (g) RT-qPCR to detect LncZFAS1 in ONFH rat femur; manifestation of data was as mean ± SD (n = 10).

**Figure 2:** Knockdown LncZFAS1 perfects ONFH in rats. (a) RT-qPCR detection of LncZFAS1 knockdown efficiency; (b) HE staining to detect the pathological changes of femur after LncZFAS1 knockdown; (c) DXA analysis to detect femoral BMD after knockdown of LncZFAS1; (d) femoral ALP after knockdown of LncZFAS1; (e) TUNEL staining to detect femoral osteocyte apoptosis after knockdown of LncZFAS1; (f) immunohistochemical detection of femoral BMP-3, BMP-9, and OCN after knockdown of LncZFAS1.

RETRACTED

**Figure 3:** Knockdown LncZFAS1 motivates osteoblast viability and bone formation. (a) CCK-8 to detect the effect of 0.1, 0.5, 1, or 5 *μ*M DEX on the viability of MC3T3-E1 cells; (b) RT-qPCR to detect LncZFAS1 knockdown efficiency; (c) CCK-8 to detect the effect of DEX treatment or knockdown LncZFAS1 on MC3T3-E1 cell viability; (d) flow cytometry to detect the effect of DEX treatment or knockdown LncZFAS1 on the apoptosis rate of MC3T3-E1 cells; (g) Western blot to detect the effect of DEX treatment or knockdown LncZFAS1 on BMP-9, BMP-3, and OCN in MC3T3-E1 cells.

**Figure 4:** LncZFAS1 competitively adsorbs miR-124-3p. (a) Bioinformatics website prediction of the potential binding sites of LncZFAS1 and miR-124-3p; (b) RT-qPCR detection of the effect of knockdown LncZFAS1 on miR-124-3p in rat femur and MC3T3-E1 cells; (c) RT-qPCR to detect the effect of knockdown LncZFAS1 on miR-124-3p in MC3T3-E1 cells; (d) the luciferase activity assay to detect the targeting relationship between LncZFAS1 and miR-124-3p; (e) RIP assay to detect the enrichment of LncZFAS1 and miR-124-3p in Ago2.

**Figure 5:** LncZFAS1 influences osteoblast viability and bone formation by modulating miR-124-3p. (a) RT-qPCR to detect miR-124-3p in MC3T3-E1 cells after cotransfection of oe-LncZFAS1 and miR-124-3p-mimic; (b) CCK-8 to detect the effect of the cotransfection of oe-LncZFAS1 and miR-124-3p-mimic on the viability of MC3T3-E1 cells; (c) flow cytometry to detect the effect of cotransfection of oe-LncZFAS1 and miR-124-3p-mimic on the apoptosis rate of MC3T3-E1 cells; (d) Alizarin red staining to detect the effect of cotransfection of oe-LncZFAS1 and miR-124-3p-mimic on the calcification ability of MC3T3-E1 cells; (e) ALP staining to detect the effect of cotransfection of oe-LncZFAS1 and miR-124-3p-mimic on ALP activity of MC3T3-E1 cells; (f) Western blot detection of the effect of cotransfection of oe-LncZFAS1 and miR-124-3p-mimic on BMP-9, BMP-3, and OCN in MC3T3-E1 cells.

**Figure 6:** MiR-124-3p targets TGFBR3. (a) Bioinformatics website prediction of the potential binding sites of TGFBR3 and miR-124-3p; (b) Western blot detection of the effect of GC on TGFBR3 in rat femurs; (c) Western blot to detect the effect of knockdown LncZFAS1 on TGFBR3 in MC3T3-E1 cells; (d) the luciferase activity assay to detect the targeting relationship between TGFBR3 and miR-124-3p; (e) RIP assay to detect the enrichment of TGFBR3 and miR-124-3p in Ago2.

**Figure 7:** Elevation of TGFBR3 depresses osteoblast viability and bone formation. (a) Western blot to detect the elevation efficiency of TGFBR3; (b) CCK-8 to detect the effect of elevation of TGFB43 on the viability of MC3T3-E1 cells; (c) flow cytometry to detect the effect of elevation of TGFB43 on the apoptosis rate of MC3T3-E1 cells; (d) Alizarin red staining to detect the effect of elevation of TGFB43 on the calcification ability of MC3T3-E1 cells; (e) ALP staining to detect the effect of elevation of TGFB43 on ALP activity of MC3T3-E1 cells; (f) Western blot to detect the effect of elevation of TGFB43 on MC3T3-E1 cellular BMP-9, BMP-3, and OCN.

RETRACTED

**Figure 8:** GCs impact osteoblast viability and bone formation by modulating the LncZFAS1/miR-124-3p/TGFBR3 axis. (a) RT-qPCR or Western blot to detect miR-124-3p and TGFBR3 in MC3T3-E1 cells after cotransfection of oe-LncZFAS1 and si-TGFBR3; (b) CCK-8 to detect the effect of the cotransfection of oe-LncZFAS1 and si-TGFBR3 on the viability of MC3T3-E1 cells; (c) flow cytometry to detect the effect of cotransfection of oe-LncZFAS1 and si-TGFBR3 on the apoptosis rate of MC3T3-E1 cells; (d) Alizarin red staining to detect the effect of cotransfection of oe-LncZFAS1 and si-TGFBR3 on the calcification ability of MC3T3-E1 cells; (e) ALP staining to detect the effect of cotransfection of oe-LncZFAS1 and si-TGFBR3 on ALP activity of MC3T3-E1 cells; (f) Western blot detection of the effect of cotransfection of oe-LncZFAS1 and si-TGFBR3 on BMP-9, BMP-3, and OCN in MC3T3-E1 cells.

**Table 1:** PCR primer sequence.

Primer sequence (5′–3′)	
LncZFAS1	F: 5′- AACCAGGCTTTGATTGAACC-3′
	R: 5′- ATTCCATCGCCAGTTTCT-3′
miR-124-3p	F: 5′- GCTTAAGGCACGCGG-3′
	R: 5′- GTGCAGGGTCCGAGG-3′
ALP	F: 5′- GGCCCAGGGCCCGGG CACCCACAAG-3′
	R: 5′- CTGGAGGCCAGAAGTGGGTTTGGCC-3′
GAPDH	F: 5′- CTGCCAACGTGTCAGTGGTG-3′ R: 5′- TCAGTGTAGCCCAGGATGCC-3′
U6	F: 5′- CGAATTTGCGTGTCATCCTT-3′
	R: 5′- CGAATTTGCGTGTCATCCTT-3′

Note: F: forward; R: reverse.

## Data Availability

The experimental data used to support the findings of this study are available from the corresponding author upon request.
